# Efficacy, Safety, and Tumor Marker Inhibition of Apatinib Combined with Conventional Chemotherapy Regimens for Patients with Advanced Triple-Negative Breast Cancer

This article has been retracted.

**DOI:** 10.1155/2021/8720679

**Published:** 2021-10-13

**Authors:** Jianzhao Chen, Lixia Feng, Qinghua Sheng, Lianna Li

**Affiliations:** Department of Pharmacy, Rizhao Central Hospital, No. 66, Wanghai Street, Rizhao City 276800, Shandong Province, China

## Abstract

**Objective:**

Triple-negative breast cancer (TNBC) is an aggressive disease with highly invasive nature and poor outcomes. Due to the absence of specific treatment strategies for this tumor subgroup, patients with TNBC are treated with conventional therapeutics, frequently leading to systemic relapse. In this study, we sought to investigate apatinib combined with conventional chemotherapy regimens in treating patients with advanced TNBC concerning the efficacy, safety, expressions of tumor markers, and patient survival.

**Methods:**

This is a prospective study including 150 cases of advanced TNBC who were randomly arranged into a conventional group and combined group, with 75 cases per group. The patients in the conventional group were treated with conventional chemotherapy, and those in the combined group were treated with apatinib combined with conventional chemotherapy. The peripheral blood was collected from each patient, and carcinoembryonic antigen (CEA), carbohydrate antigen 153 (CA153), and carbohydrate antigen 125 (CA125) were determined. The expressions of nuclear proliferation antigen marker (Ki67), *β*-catenin, and E-cadherin were determined in the biopsy collected from each patient.

**Results:**

The objective remission rate (ORR) and disease control rate (DCR) (41.33% and 81.33%) in the combined group were notably higher than those in the conventional group (29.33% and 68.00%) (*P* < 0.05). After treatment, the serum levels of CEA, CA153, and CA125 and the expressions of Ki67 and *β*-catenin were declined, but the expression of E-cadherin was increased in both groups; the combined group exhibited lower serum levels of CEA, CA153, and CA125, and the expressions of Ki67 and *β*-catenin were concurrent with a higher expression of E-cadherin than the conventional group (*P* < 0.05). No significant difference was noted between the two groups regarding the occurrence of adverse reactions (*P* > 0.05). Improved progression-free survival (PFS) was observed in the combined group compared to the conventional group (*P* < 0.05.

**Conclusion:**

These findings suggest that apatinib combined with conventional chemotherapy regimens confers a prolonged PFS for treating patients with advanced TNBC.

## 1. Introduction

Triple-negative breast cancer (TNBC) represents a particularly aggressive subtype of BC that is characterized by high heterogeneity, aggressive nature, high metastatic potential, proneness to relapse, and poor prognosis due to a lack of estrogen receptor (ER), progesterone receptor (PR), or human epidermal growth factor receptor 2 (HER-2) [1]. TNBC has been identified with six distinct TNBC subtypes, each of which exhibits a unique molecular signature, leading to different prognoses and possibly various responses to therapy [2]. TNBC accounts for 15% to 20% of BC cases, and the median survival for women with metastatic TNBC is less than 12 months [3, 4]. TNBC typically occurs in younger people (<40 years) who are more African American and have shorter progression-free survival (PFS) and overall survival (OS) compared to non-TNBC patients [5, 6]. Due to no response or long-term availability to endocrine therapy or HER-2 treatment, patients with TNBC are treated with conventional chemotherapy regimens including platinum and paclitaxel and standardized TNBC treatment regimens are still lacking [7, 8]. At present, two PARP inhibitors (olaparib and talazoparib), anti-PD-L1 monoclonal antibody (atezolizumab) and an antibody drug conjugate targeting Trop-2 (sacituzumab govitecan-hziy) have been approved in select subpopulations of patients with metastatic TNBC [9–11]. On the other hand, there are primary research with investigation of radiosensitization with combined use of olaparib and PI-103 in TNBC and even a clinical trial investigating the efficacy and safety of targeted drugs combined with radiotherapy in patients with metastatic TNBC [12, 13]. However, PFS of patients with advanced TNBC remains still unsatisfactory or to be confirmed.

Substantial evidence demonstrated the important role of angiogenesis played in the occurrence and development of tumors, and registered tyrosine kinase inhibitors targeting vascular endothelial growth factor (VEGF) could attenuate angiogenesis [14]. Apatinib, a tyrosine kinase inhibitor, can specifically inhibit vascular endothelial growth factor receptor 2 (VEGFR-2) and is the second antiangiogenic drug to be approved in China (Aitan®) for the treatment of advanced or metastatic gastric cancer [15]. Moreover, its clinical use to treat chemotherapy-experienced patients with advanced gastric cancer or other advanced cancers such as gynecological cancers, hepatocellular carcinoma, non-small-cell lung cancer, breast cancer, thyroid cancer, and sarcomas was often assessed. More interesting, apatinib was assessed in combination with anti-PD-1 antibody for treating advanced human cancers in clinical trials [16, 17]. However, the use of apatinib as subsequent-line treatment in Chinese patients with other advanced or metastatic solid tumours, such as TNBC, is supported by limited evidence. Therefore, this prospective study including 150 cases of advanced TNBC, and all of them were randomly arranged into a conventional group and combined group, with 75 cases per group. The patients in the conventional group were treated with conventional chemotherapy, and those in the combined group were treated with apatinib combined with conventional chemotherapy. We sought to investigate apatinib combined with conventional chemotherapy regimens in treating patients with advanced TNBC concerning the efficacy, safety, expressions of tumor markers, and patient survival.

## 2. Materials and Methods

### 2.1. Study Design

A total of 150 patients with advanced TNBC were diagnosed and treated in our hospital from June 2016 to November 2018, and all of them fulfill predefined inclusion criteria: diagnosis confirmed by pathology and cytology, negative for ER and PR by immunohistochemistry, and negative for HER-2 by fluorescence in situ hybridization; with an estimated survival time of more than 3 months; aged more than 18 years with complete clinical data; the presence of at least one detectable lesion; signed the informed consent form; and study design meets the *Declaration of Helsinki*. Exclusion criteria: contraindication to chemotherapy; severe heart, lung, and kidney dysfunction; mental illness; the presence of other malignancies; acute cerebral infarction, serious arrhythmia, heart failure, and other major cardiovascular diseases; undergoing thrombolytic or anticoagulant therapy; hypertension out of control by single antihypertensive treatment; allergic to study drug; poor medication compliance; difficult to determine the efficacy of drugs due to radiotherapy, immunotherapy, or other targeted therapy; withdrawal from the study or lost to follow-up; and lactation or pregnancy. The study was approved by the Ethics Committee of Rizhao Central Hospital.

### 2.2. Treatment Protocols

All patients were given required examinations after admission and received conventional chemotherapeutic regimes, including 135–175 mg/m^2^ paclitaxel (specification: 30 mg, approval No. gyzz h20178012, Guangdong Xinghao Pharmaceutical Co., Ltd., China), 60 mg/m^2^ epirubicin (specification: 10 mg, approval No. gyzz h20123260, Shandong Xinshidai Pharmaceutical Co., Ltd., China), and 8 mg ondansetron (specification: 4 mg, approval No. gyzz h10960146, Fuan Pharmaceutical Group Ningbo Tianheng Pharmaceutical Co., Ltd., China) on the first day at their admission according to the doctor's advice, twice a day, 21 days/cycle.

Those arranged into the combined group were additionally treated with apatinib tablets (specification: 10 tablets each for 0.25 g, approval No. gyzz h20140103, Jiangsu Hengrui Pharmaceutical Co., Ltd., China) orally, with an initial dose of 500 mg/time, once a day, 21 days/cycle. The investigator can appropriately reduce the initial dose to 425 mg/day, 21 days/cycle, according to specific situations.

### 2.3. Adverse Reactions and Follow-Up

In case of grade III-IV hematological and nonhematological adverse reactions during the treatment, the administration and dose adjustment can be delayed. The treatment course of patients in the two groups is ≥2 cycles until the imaging examination indicated the progress of the patient's condition, or the administration is terminated. All patients received CT or MRI to evaluate the curative effect at the end of every 2 cycles. The patients were followed up for 12 months by telephone and door-to-door visit.

### 2.4. Peripheral Blood Collection and Serum Extraction

Before treatment and the second cycles of chemotherapeutic regimes, 5 ml of fasting elbow venous blood was taken from each patient in the morning. After centrifugation at 3500 r/min for 10 min, the supernatant was immediately stored it in a low-temperature refrigerator at −20°C for further testing. The levels of serum CEA, CA153, and CA125 were detected by using an Abbott I2000 SR automatic chemiluminescence analyzer (Architect, IL, USA).

### 2.5. Immunohistochemistry

The immunohistochemical staining of nuclear associated antigen markers (Ki67), E-cadherin, and *β*-catenin in the lesion biopsy tissues was analyzed. Before treatment and the second cycles of chemotherapeutic regimes, color ultrasound-guided fine needle biopsy, with outer diameter 2 mm, was performed to obtain breast lesion tissues. After formaldehyde fixation, gradient elution with ethanol, xylene treatment, and paraffin-embedding, the tissues were then sectioned (thickness 4 *μ*m) and mounted onto the slides. After deparaffinization and antigen retrieval, the sections were blocked and incubated with primary antibodies to Ki67 (ab16667, Abcam, UK), E-cadherin (ab40772, Abcam), and *β*-catenin (ab32572, Abcam) in strict accordance with the procedures listed in the kit's instructions. The staining was observed and evaluated by two professional doctors in double-blind. The cumulative optical density of fields of view was calculated by Image Pro Plus 6.0 software.

### 2.6. Outcome Measures

1. The clinical effects of the two groups were compared. At the end of the second cycles of chemotherapeutic regimes, the lesions were measured in all patients, and CT or MRI evaluation was performed. The Response Evaluation Criteria in Solid Tumors (RECIST) provides a simple and pragmatic methodology to evaluate the activity and efficacy of new cancer therapeutics in solid tumors [6], which is classified into complete remission (CR) and partial remission (PR), disease stability (SD), and disease progression (PD). CR is defined when all target lesions disappear; PR is defined when comprehensive reduction of baseline lesion length ≥30% is observed; PD is defined when new lesions appear or the total length of baseline lesions is increased by more than 20% by 1 cm; SD is defined when the sum of baseline long menstrual length of lesions is decreased but fails to reach PR or the sum of baseline long menstrual length of lesions is increased but fails to reach PD. Objective response rate (ORR) consisted of CR + PR, and disease control rate (DCR) consisted of CR + PR + SD.
2. The levels of serum CEA, CA153, and CA125 were compared between the two groups before treatment and at the end of the second cycle. Normally, the CA125 level should be less than 35 U/mL, the CEA level less than 5 ng/ml, and the CA153 level less than 25 U/ml.
3. The expression levels of Ki67, E-cadherin, and *β*-catenin in the lesion biopsy tissues were compared between the two groups before treatment and at the end of the second cycle.
4. The adverse reactions of the two groups were commonly graded from 0 to IV according to World Health Organization (WHO)/NCI criteria for toxic and side effects of chemotherapy drugs [7].
5. The PFS from study recruitment to tumor progression or death was compared between the two groups after 12-month follow-up.

### 2.7. Statistical Analysis

All data in this study were analyzed by SPSS21.0 software. The measurement data were described as a manner of mean ± standard deviation and analyzed by the *t*-test. The count data were described as a manner of ratio and analyzed by the chi-square test. The Kaplan–Meier method was used to plot the PFS of the two groups, and differences between curves were analyzed by the log-rank test. Inspection levels of *α* = 0.05 and *P* < 0.05 indicate the presence of a statistically significant difference.

## 3. Results

A total of 150 patients were randomly arranged into the conventional group and combined group. The conventional group (*n* = 75): all women, aged from 22 to 78 years, with an average of (47.17 ± 5.27) years; 47 cases were postmenopausal, and 28 cases were premenopausal; pathological classification: 6 cases of simple carcinoma, 62 cases of invasive ductal carcinoma, and 7 cases of myeloid carcinoma; and metastatic sites: lung metastasis in 30 cases, liver metastasis in 14 cases, bone metastasis in 20 cases, and lymph node metastasis in 11 cases. The combined group (*n* = 75): all women, aged 28–79 years, with an average of (47.24 ± 5.16) years; 46 cases were postmenopausal, and 29 cases were premenopausal; pathological classification: 8 cases of simple carcinoma, 60 cases of invasive ductal carcinoma, and 7 cases of myeloid carcinoma; and metastatic sites: lung metastasis in 32 cases, liver metastasis in 13 cases, bone metastasis in 18 cases, and lymph node metastasis in 12 cases. The two groups were comparable considering no significant difference on age, menopausal status, pathological classification, and metastatic sites (*P* > 0.05).

The clinical efficacy of conventional chemotherapy alone or combined with apatinib was evaluated using the RECIST after at least 2 cycles. There was no treatment-related death occurring. ORR and DCR in the combined group were 41.33% and 81.33%, respectively, which were significantly higher than those in the conventional group, 29.33% and 68.00%, respectively (*P* < 0.05, Table 1).

The serum levels of CEA, CA153, and CA125 in the conventional group and combined group were declined significantly after at least 2 cycles (*P* < 0.05). The levels of serum CEA, CA153, and CA125 in the combined group were significantly lower than those in the conventional group (*P* < 0.05, Table 2).

After at least 2 cycles of treatment, the expression levels of Ki67 and *β*-catenin were decreased and the expression level of E-cadherin was increased in the conventional group and combined group (*P* < 0.05). The expression levels of Ki67 and *β*-catenin were lower and the expression level of E-cadherin was higher in the combined group than those in the conventional group (*P* < 0.05, Table 3).

The main adverse reactions of grade I-II in the two groups were bone marrow suppression (neutropenia and leucopenia), pain and gastrointestinal reaction, and the serious adverse reactions of grade III-IV were gastrointestinal reaction, hypertension, and bone marrow suppression. There was no significant difference in the incidence rate of grade I-II adverse reactions and grade III-IV serious adverse reactions between the conventional group and combined group (*P* > 0.05, Table 4).

All patients were followed up at the end of the second cycles of chemotherapeutic regimes. The follow-up time was 12 months, and the median follow-up time was 5 months. The median follow-up time was 5.5 months in the combined group and 3.5 months in the conventional group. The median PFS of the conventional group was 2.7 months, and the median PFS of the combined group was 5.6 months. The PFS in the combined group was significantly longer than that in the conventional group (*P* < 0.05, Figure 1).

## 4. Discussion

At present, the treatment of TNBC has entered the era of individualized treatment based on molecular typing, and targeted therapy plays extremely important roles [18]. In this study, we performed prospective study and recruited 150 cases of advanced TNBC who were randomly arranged into a conventional group and combined group, with 75 cases per group. The patients in the combined group were given oral administration of apatinib followed by conventional chemotherapy regimens and exhibited prolonged PFS.

Apatinib is the first small-molecule antiangiogenesis targeted drug approved for its safety and efficacy in advanced gastric cancer worldwide [19]. It is also a single drug that significantly prolongs the survival time after the failure of standard chemotherapy for advanced gastric cancer. At the same time, this drug is the only oral preparation among targeted drugs for gastric cancer, which can effectively improve the treatment compliance of patients and significantly reduce treatment costs [20]. Apatinib functions by highly selective competition for ATP binding sites of intracellular VEGFR-2, blocking downstream signal transduction, and inhibiting neoangiogenesis in tumor tissues [21]. In this study, included TNBC patients received at least 2 cycles of treatment protocols, and no deaths occurred after treatment. The median follow-up time in the combined group was 5.5 months. ORR and DCR were 41.33% and 81.33%, respectively, which were significantly better than those in the conventional group. The results show that oral administration of apatinib followed by conventional chemotherapy regimens can effectively control the disease progression and prolong the survival time of TNBC patients. In a multicenter phase II study conducted by Hu et al., they recruited 59 patients with metastatic TNBC and demonstrated an apatinib dose of 500 mg rather than 750 mg is the recommended starting dose for the heavily pretreated metastatic TNBC patients with measurable rate of PR and PFS [22].

The detection method of tumor markers is simple, rapid, and minimally invasive, which plays an important role in the diagnosis, clinical efficacy, and prognosis of BC [23]. The American Society of Clinical Oncology recommends peripheral blood tumor markers such as CA153, CA125, and CEA as routine detection for BC diagnosis and prognosis [24, 25]. CA153 has been first discovered in BC cells, which is a variant of glycoprotein in the epithelial cells of BC [26]. CA125 is a major tumor marker of ovarian cancer. However, a large number of clinical studies have confirmed that CA125 has increased in BC subtypes [27]. CEA is elevated remarkably in a variety of malignant tumors and is a broad-spectrum tumor marker [28]. In this study, after treatment, the combined group exhibited lower serum levels of CEA, CA153, and CA125 than the conventional group, suggesting the additional oral administration of apatinib could enhance the antitumor effects of conventional chemotherapy for patients with advanced TNBC.

Malignant tumor cells are characterized by uncontrolled cell proliferation caused by aberrant cell cycle progression, which is also one of the biggest characteristics different from benign tumors [29]. In this study, the expressions of Ki67, *β*-catenin, and E-cadherin in the lesion tissue were analyzed before and after treatment. Ki67 is currently one of the most reliable indicators for clinical detection of tumor cell proliferation activity [30], including for BC. In the advanced refractory BC patients, an increased expression level of Ki67 reflects enhanced tumor cell proliferation. In this condition, the tumor cells are more vulnerable to invasion and metastasis to the liver, bone, and lymph nodes [31]. E-cadherin is a member of the calcium adhesion family and plays an important role in maintaining cell polarity and intercellular adhesion. Its low expression in tumor tissues often indicates the tumor cells with high invasiveness [32]. According to the study performed by Tavakolian et al., the expression level of E-cadherin in BC tissue is significantly lower than that in adjacent tissues, and the expression level of E-cadherin is correlated with the survival time of BC [33]. *β*-Catenin is one of the downstream factors of the Wnt pathway. The Wnt signal is deactivated in normal mature cells, and the content of *β*-catenin is very low in the cytoplasm. When breast cells become aggressive, the degradation *β*-catenin is impaired and more *β*-catenin aggregates into the nucleus, which activates the transcription of downstream target genes and leads to cancer initiation [34]. The results of this study showed the expression levels of Ki67 and *β*-catenin were lower and the expression level of E-cadherin was higher in the combined group than those in the conventional group, indicating apatinib could reduce the expressions of Ki67, E-cadherin, and *β*-catenin in the lesion.

In conclusion, the study provides evidence that additional oral administration of apatinib during conventional chemotherapy regimens confers a prolonged PFS for treating patients with advanced TNBC, which also could reduce serum CEA, CA153, and CA125 levels, and inhibiting tumor progression. Further clinical experience with a larger sample size and more comprehensive longitudinal gene detection analysis and long-term pharmacovigilance data would be warrant to more definitively validate the efficacy and safety profile of apatinib, including its use in combination with conventional chemotherapy agents for treating advanced TNBC.

## Figures and Tables

**Figure 1:** Kaplan–Meier curves of PFS between the conventional and combined groups after treatment.

**Table 1:** The clinical efficacy between the conventional and combined groups after treatment.

Group	CR	PR	SD	PD	ORR	DCR
Conventional (*n* = 75)	2 (2.67%)	20 (26.67%)	29 (38.671%)	24 (32.00%)	22 (29.33%)	51 (68.00%)
Combined (*n* = 75)	6 (8.00%)	25 (33.33%)	30 (40.00%)	14 (18.67%)	31 (41.33%)^a^	61 (81.33%)^a^

^a^ *P* < 0.05 compared with the conventional group.

**Table 2:** The serum levels of CEA, CA153, and CA125 between the conventional and combined groups before and after treatment.

Time	Group	CEA (ng/ml)	CA153 (U/ml)	CA125 (U/ml)
Before	Conventional (*n* = 75)	54.56 ± 5.52	55.14 ± 5.05	154.33 ± 16.85
	Combined (*n* = 75)	54.29 ± 6.43^b^	56.37 ± 5.48^b^	155.94 ± 15.57^b^
*t*		0.171	0.482	0.726
*P*		0.271	0.119	0.094
After	Conventional (*n* = 75)	33.46 ± 4.03^a^	38.12 ± 3.06^a^	67.91 ± 5.87^a^
	Combined (*n* = 75)	20.14 ± 3.04^ab^	22.19 ± 1.10^ab^	24.65 ± 3.99^ab^
*t*		7.184	8.016	7.253
*P*		0.001	0.001	0.001

^a^ *P* < 0.05 for comparison in the same group before and after treatment; ^b^*P* < 0.05 compared with the conventional group.

**Table 3:** The serum expression levels of Ki67, E-cadherin, and *β*-catenin between the conventional and combined groups before and after treatment.

Time	Group	Ki67	E-cadherin	*β*-Catenin
Before	Conventional (*n* = 75)	112.83 ± 10.65	74.01 ± 6.57	131.18 ± 14.72
	Combined (*n* = 75)	111.92 ± 10.76	74.21 ± 6.34	131.18 ± 14.22
*t*		0.175	0.271	0.162
*P*		0.872	0.719	0.804
After	Conventional (*n* = 75)	82.26 ± 6.49^a^	85.49 ± 6.47^a^	120.01 ± 8.38^a^
	Combined (*n* = 75)	57.82 ± 5.36^ab^	102.81 ± 7.73^ab^	101.15 ± 5.72^ab^
*t*		8.213	7.982	9.092
*P*		0.001	0.001	0.001

^a^ *P* < 0.05 for comparison in the same group before and after treatment; ^b^*P* < 0.05 compared with the conventional group.

**Table 4:** The occurrence rate of adverse reactions between the conventional and combined groups after treatment.

Adverse reaction	Group	Neutropenia	Leukocytopenia	Pain	Gastrointestinal reaction	Hypertension	Weakness	Oral mucositis	Hand-foot syndrome
Grade I-II	Conventional (*n* = 75)	22	35	34	35	22	33	16	26
	Combined (*n* = 75)	22	34	30	33	21	31	13	25
*χ* ^2^		1.515	1.194	1.175	1.216	1.271	1.073	1.056	1.162
*P*		0.171	0.186	0.272	0.248	0.319	0.215	0.137	0.104
Grade III-IV	Conventional (*n* = 75)	7	0	9	17	16	2	4	3
	Combined (*n* = 75)	8	1	8	16	17	3	5	3
*χ* ^2^		1.115	1.074	1.213	1.072	1.082	1.061	1.077	1.092
*P*		0.215	0.218	0.191	0.143	0.162	0.214	0.117	0.241

## Data Availability

The data used for this study are included in the article.

## References

[1] Yin L., Duan J.-J., Bian X.-W., Yu S.-c. (2020). Triple-negative breast cancer molecular subtyping and treatment progress. *Breast Cancer Research*.

[2] Sporikova Z., Koudelakova V., Trojanec R., Hajduch M. (2018). Genetic markers in triple-negative breast cancer. *Clinical Breast Cancer*.

[3] Loibl S., Poortmans P., Morrow M., Denkert C., Curigliano G. (2021). Breast cancer. *The Lancet*.

[4] Abramson V. G., Lehmann B. D., Ballinger T. J., Pietenpol J. A. (2015). Subtyping of triple-negative breast cancer: implications for therapy. *Cancer*.

[5] Liedtke C., Hess K. R., Karn T. (2013). The prognostic impact of age in patients with triple-negative breast cancer. *Breast Cancer Research and Treatment*.

[6] Bauer K. R., Brown M., Cress R. D., Parise C. A., Caggiano V. (2007). Descriptive analysis of estrogen receptor (ER)-negative, progesterone receptor (PR)-negative, and HER2-negative invasive breast cancer, the so-called triple-negative phenotype. *Cancer*.

[7] Keenan T. E., Tolaney S. M. (2020). Role of immunotherapy in triple-negative breast cancer. *Journal of the National Comprehensive Cancer Network*.

[8] Denkert C., Liedtke C., Tutt A., von Minckwitz G. (2017). Molecular alterations in triple-negative breast cancer-the road to new treatment strategies. *The Lancet*.

[9] Loibl S., O’Shaughnessy J., Untch M. (2018). Addition of the PARP inhibitor veliparib plus carboplatin or carboplatin alone to standard neoadjuvant chemotherapy in triple-negative breast cancer (BrighTNess): a randomised, phase 3 trial. *The Lancet Oncology*.

[10] Robson M. E., Tung N., Conte P. (2019). OlympiAD final overall survival and tolerability results: olaparib versus chemotherapy treatment of physician’s choice in patients with a germline BRCA mutation and HER2-negative metastatic breast cancer. *Annals of Oncology*.

[11] Bardia A., Mayer I. A., Vahdat L. T. (2019). Sacituzumab govitecan-hziy in refractory metastatic triple-negative breast cancer. *New England Journal of Medicine*.

[12] Jang N. Y., Kim D. H., Cho B. J. (2015). Radiosensitization with combined use of olaparib and PI-103 in triple-negative breast cancer. *BMC Cancer*.

[13] Ho A. Y., Barker C. A., Arnold B. B. (2020). A phase 2 clinical trial assessing the efficacy and safety of pembrolizumab and radiotherapy in patients with metastatic triple‐negative breast cancer. *Cancer*.

[14] Qin S., Li A., Yi M., Yu S., Zhang M., Wu K. (2019). Recent advances on anti-angiogenesis receptor tyrosine kinase inhibitors in cancer therapy. *Journal of Hematology & Oncology*.

[15] Scott L. J. (2018). Correction to: apatinib: A review in advanced gastric cancer and other advanced cancers. *Drugs*.

[16] Xu J., Zhang Y., Jia R. (2019). Anti-PD-1 antibody SHR-1210 combined with apatinib for advanced hepatocellular carcinoma, gastric, or esophagogastric junction cancer: an open-label, dose escalation and expansion study. *Clinical Cancer Research*.

[17] Zhao S., Ren S., Jiang T. (2019). Low-dose apatinib optimizes tumor microenvironment and potentiates antitumor effect of PD-1/PD-L1 blockade in lung cancer. *Cancer immunology research*.

[18] Azim H. A., Ghosn M., Oualla K., Kassem L. (2020). Personalized treatment in metastatic triple‐negative breast cancer: the outlook in 2020. *Breast Journal*.

[19] Roviello G., Ravelli A., Fiaschi A. I. (2016). Apatinib for the treatment of gastric cancer. *Expert Review of Gastroenterology & Hepatology*.

[20] Chen H.-D., Zhou J., Wen F. (2017). Cost-effectiveness analysis of apatinib treatment for chemotherapy-refractory advanced gastric cancer. *Journal of Cancer Research and Clinical Oncology*.

[21] Gao Z., Shi M., Wang Y., Chen J., Ou Y. (2019). Apatinib enhanced anti-tumor activity of cisplatin on triple-negative breast cancer through inhibition of VEGFR-2. *Pathology, Research & Practice*.

[22] Hu X., Zhang J., Xu B. (2014). Multicenter phase II study of apatinib, a novel VEGFR inhibitor in heavily pretreated patients with metastatic triple-negative breast cancer. *International Journal of Cancer*.

[23] Tozzoli R., D’;Aurizio F., Falcomer F., M.M. Basso S., Lumachi F. (2016). Serum tumor markers in stage I-II breast cancer. *Medicinal Chemistry*.

[24] Wang W., Xu X., Tian B. (2017). The diagnostic value of serum tumor markers CEA, CA19-9, CA125, CA15-3, and TPS in metastatic breast cancer. *Clinica Chimica Acta*.

[25] Zhao S., Mei Y., Wang Y., Zhu J., Zheng G., Ma R. (2015). Levels of CEA, CA153, CA199, CA724 and AFP in nipple discharge of breast cancer patients. *International Journal of Clinical and Experimental Medicine*.

[26] Tang S., Wei L., Sun Y. (2016). CA153 in breast secretions as a potential molecular marker for diagnosing breast cancer: a meta analysis. *PLoS One*.

[27] Li J., Liu L., Feng Z. (2020). Tumor markers CA15-3, CA125, CEA and breast cancer survival by molecular subtype: a cohort study. *Breast Cancer*.

[28] Tsang J. Y. S., Kwok Y. K., Chan K. W. (2013). Expression and clinical significance of carcinoembryonic antigen-related cell adhesion molecule 6 in breast cancers. *Breast Cancer Research and Treatment*.

[29] Cai Z., Liu Q. (2017). Cell cycle regulation in treatment of breast cancer. *Advances in Experimental Medicine & Biology*.

[30] Mannell A. (2016). The role of Ki-67 in breast cancer. *South African Journal of Surgery*.

[31] Dowsett M., Nielsen T. O., A’Hern R. (2011). International Ki-Assessment of Ki67 in breast cancer: recommendations from the international Ki67 in breast cancer working group. *JNCI Journal of the National Cancer Institute*.

[32] Corso G., Figueiredo J., De Angelis S. P. (2020). E‐cadherin deregulation in breast cancer. *Journal of Cellular and Molecular Medicine*.

[33] Tavakolian S., Goudarzi H., Faghihloo E. (2019). E-cadherin, Snail, ZEB-1, DNMT1, DNMT3A and DNMT3B expression in normal and breast cancer tissues. *Acta Biochimica Polonica*.

[34] Zhang Y., Wang X. (2020). Targeting the Wnt/*β*-catenin signaling pathway in cancer. *Journal of Hematology & Oncology*.

